The article "Metformin Synergizes with PD-L1 Monoclonal Antibody Enhancing Tumor Immune Response in Treating Non-Small Cell Lung Cancer and Its Molecular Mechanism Investigation" was retracted in 2023. Reasons: unreliable results or conclusions; concerns about the data; concerns about the peer review; concerns about the citations.

# Metformin Synergizes with PD-L1 Monoclonal Antibody Enhancing Tumor Immune Response in Treating Non-Small Cell Lung Cancer and Its Molecular Mechanism Investigation

**DOI:** 10.1155/2022/5983959

**Published:** 2022-09-25

**Authors:** Yifan Wang, Jingguo Hu, Yu Sun, Bo Song, Yan Zhang, Yusong Lu, Haitao Ma

**Affiliations:** ^1^The First Affiliated Hospital of Soochow University, Department of Thoracic Surgery, Suzhou 215006, China; ^2^Affiliated Hospital of Chengdu University, Department of Thoracic Surgery, Chengdu 610081, China

## Abstract

Despite non-small cell lung cancer (NSCLC) treatment is proved to be effective using PD-L1 monoclonal antibody (PD-L1 MAb), it is commonly seen in immune-related adverse events reported. We aimed to explore metformin synergized with PD-L1 MAb in treating NSCLC and its potential molecular mechanism. In mice, the transplantable lung cancer models were established and a co-culture system of CD8+T cells and LLC cells was constructed. The anti-tumor effect was assessed by xenograft tumor growth, proliferation signal Ki67 expression, and MTT assays. Immunohistochemistry and western blot assays were also conducted to determine tumor immune response as well as mechanism investigation. The results indicated that tumor volume and cell proliferation were markedly inhibited following metformin synergized with PD-L1 MAb which was more effective than either single metformin or PD-L1 MAb. The cytokines TNF-*α*, IL-2, and IFN-*γ* secretion in CD8+ T cells was significantly increased, and the immune response was enhanced by metformin synergized with PD-L1 MAb. Further, the WB results implied that metformin synergized with PD-L1 MAb could activate the AMPK pathway and inhibit mTOR. AMPK inhibitor (Compound C) was added, and the results showed that the anti-tumor effect was reduced in metformin + PD-L1 MAb + CC than in metformin + PD-L1 MAb which indicates the metformin synergized with PD-L1 MAb efficacy was AMPK pathway dependent. In conclusion, metformin synergized with PD-L1 MAb has better efficacy against NSCLC than metformin or PD-L1 MAb alone in an AMPK-dependent way and facilitates increasing CD8+ T cell infiltration and enhancing tumor immune response.

## 1. Introduction

According to the World Health Organization statistics, the leading cause of death worldwide remains cancers in 2020, causing about 10 million deaths. In terms of new cancer cases, breast, lung, and colorectal cancers were the most common types of cancers in 2020. Lung cancer caused the most deaths, with about 1.8 million deaths, followed by colorectal cancer and liver cancer (935,000 and 830,000). Lung cancer has been recognized as one of the recent top diseases with high morbidity and fatality. There is still no effective treatment for advanced lung cancer whose clinical treatment still faces huge challenges, with a 5-year survival rate as low as 5% [1]. Lung cancer has been divided into small cell lung cancer (SCLC) and non-small cell lung cancer (NSCLC). The latter takes up nearly 85% of cases with lung cancer [2]. There are three types of NSCLC: adenocarcinoma, which accounts for 40% of all NSCLC diagnoses, squamous cell carcinoma, approximately 25% to 30% and the third one is large cell carcinoma, which is rare at around 10%–15% of the diagnosed cases [3].

The article "Metformin Synergizes with PD-L1 Monoclonal Antibody Enhancing Tumor Immune Response in Treating Non-Small Cell Lung Cancer and Its Molecular Mechanism Investigation" was retracted in 2023. Reasons: unreliable results or conclusions; concerns about the data; concerns about the peer review; concerns about the citations.

The therapy options of SCLC include surgical excision, radiation therapy, chemical therapy, immunotherapy, and targeted therapy based on different stages of the disease diagnosed. Due to most patients being in advanced stages when the disease is diagnosed, the treatment options are limited, mostly systemic radiotherapy, supplemented by chemotherapy. For those sensitive to gene mutations, targeted therapy can be employed, but large toxic side effects and drug resistance have existed. Therefore, the treatment effect is not good, and it is difficult to effectively improve patients' survival rate. In recent years, tumor immunotherapy research has obtained rapid progress. Clinical studies have found that programmed death ligand 1 (PD-L1)/programmed cell death (PD-1) can enhance the resistance of the tumor microenvironment to the body's normal immunity by inhibiting immune response, promoting immune escape, and other mechanisms. PD-1 and PD-L1 have become new immunotherapeutic targets, and breakthroughs are made in NSCLC treatment in multiple clinical trials [4, 5]. As the main ligand of PD-1, PD-L1 is currently recognized as a negative immunoregulatory protein and is highly expressed in many malignant tumors, including NSCLC [6, 7], melanoma [8], renal cell carcinoma [9], prostate cancer [10], breast cancer [11]. Highly expressed PD-L1 in NSCLC links to high tumor aggressiveness and poor prognosis [12, 13].

Metformin is a safe oral biguanide drug. EVANS et al. found that metformin is associated with reduced tumor prevalence for diabetic patients, and its possible anti-tumor effect has attracted widespread attention [14]. It also retards cell proliferation, migration, and invasion of tumors as well as induces cell apoptosis. The anti-tumor effect involves multiple genes and signaling pathways. Metformin can activate the adenosine monophosphate-activated protein kinase (AMPK) pathway or directly inhibit the mammalian target of the rapamycin (mTOR) pathway. AMPK can activate the catabolic pathway in tissue cells and inhibit the anabolic pathway, which fundamentally reduces the generation of tumor cell energy and inhibits tumor cell proliferation. As a serine-threonine protein kinase, mTOR regulates tumor cell survival, proliferation, invasion, and metastasis by activating ribosomal kinases in the downstream of PI3K/Akt pathway. Currie et al. revealed that metformin application can minimize the risk of getting lung cancer [15]. Furthermore, the study also revealed that metformin can improve lung cancer patients' survival rate at stage IV complicated with diabetes mellitus [16]. Patients with type 2 diabetes can also benefit from it with a lower risk of lung cancer [17], and effectively prevent lung cancer caused by tobacco carcinogens [18]. Studies have also demonstrated that metformin reverses epithelial-mesenchymal transition and suppresses the growth of lung adenocarcinoma [19], and enhances the sensitivity of radiotherapy in A549, H1299, and SK-MES lung cancer cell lines [20]. Additional chemotherapeutic medications could strengthen the cytotoxic effect of chemotherapeutic drugs, inhibit the growth of tumor stem cells, and reverse platinum drug resistance [21, 22].

The article "Metformin Synergizes with PD-L1 Monoclonal Antibody Enhancing Tumor Immune Response in Treating Non-Small Cell Lung Cancer and Its Molecular Mechanism Investigation" was retracted in 2023. Reasons: unreliable results or conclusions; concerns about the data; concerns about the peer review; concerns about the citations.

Some studies have found that metformin exerts its anti-tumor effect mainly by affecting PD1/PD-L1 and T lymphocytes. Therefore, this study explored the effect of metformin synergized with PD-L1 monoclonal antibody (PD-L1 MAb) in treating NSCLC at the animal level by constructing a subcutaneous transplanted tumor model of lung cancer. CD8+ T cells were collected from mice, Lewis lung cancer (LLC) cells were purchased, and a co-culture system of both CD8+ T and LLC cells was constructed for the investigation of efficacy and molecular mechanism of metformin synergized with PD-L1 MAb against NSCLC treatment. This provides an alternative drug treatment for NSCLC and a theoretical basis for the treatment of NSCLC patients with metformin synergized with PD-L1 MAb clinically.

## 2. Materials and Methods

### 2.1. Animal Model

Twenty-four SPF Balb/*c* mice (6–8 w, body weight 20 ± 5 g) were purchased from Chongqing Byrness Weil biotech Ltd. Animal experiment protocol was approved by the First Affiliated Hospital of Soochow University. Adapted to feeding for 7 days in an animal room with indoor temperature (23 ± 2)°C, relative humidity of 60%, and 12 h day-night cycle lighting, they were classified into four groups randomly with six in each group. The animals were inoculated with 170 *μ*L (1 × 10^7^/mL) lung cancer LLC cells (Type Culture Collection, Chinese Academy of Sciences) to establish a mouse model of lung cancer subcutaneously transplanted tumor.

### 2.2. Administration of Medicine

On the 8th day after the successful inoculation of the transplanted tumor, the metformin treatment group was given metformin (200 mg/kg) in drinking water, and the PD-L1 MAb group was intraperitoneally injected with 200 *μ*g PD-L1 MAb (Sigma), once every 3 days. The metformin + PD-L1 MAb group was given metformin (oral) and intraperitoneal injection of PD-L1 MAb, and the control group was injected with an equal quantity of normal saline. Thirty days later, all animals were anesthetized with 30 mg/kg pentobarbital sodium and then put to death, and the tumor tissue was removed and embedded for subsequent experiments.

The article "Metformin Synergizes with PD-L1 Monoclonal Antibody Enhancing Tumor Immune Response in Treating Non-Small Cell Lung Cancer and Its Molecular Mechanism Investigation" was retracted in 2023. Reasons: unreliable results or conclusions; concerns about the data; concerns about the peer review; concerns about the citations.

### 2.3. Western Blotting

Total protein was obtained by RIPA lysis buffer. Bicinchoninic acid (BCA) was used to quantify the protein, then the protein was denatured at 100°C for 6 min. Protein electrophoresis was performed in 13% SDS-polyacrylamide gel. A PVDF membrane was applied for protein transfer and sealed with skim milk for 1 h. Following three cycles of washing with TBST, 5 min of each, primary antibody (1 : 1000) was added for incubation overnight at 4°C. A cycle of washing was conducted with TBST again, and a secondary antibody (1 : 2000) was supplied for culture at 37°C for 1 h. Chemiluminescence color was exposed and collected following TBST washing [23]. Primary antibodies were purchased from abclonal: anti-p-AMPK (A12491), anti-mTOR (A2445), anti-Ki67 (A2094), and anti-*β*-Actin (AC026).

### 2.4. Immunohistochemistry

The tumor tissues of mice in all groups were obtained, fixed with a 4% paraformaldehyde agent, and processed into paraffin-embedded sections. The paraffin blocks of representative tumor areas of mice were cut into 4 *μ*m sections for staining. After dissociation and hydration, deparaffinization, rehydration and antigen retrieval, endogenous peroxidase activity was quenched using 3% hydrogen peroxide via incubation in the dark at room temperature for 15 min, followed by PBS washing three times for antigen retrieval. The sections were incubated overnight with rabbit anti-mouse CD8 antibody (1 : 100), washed three times on a shaker, and then added secondary antibody and incubated at room temperature for 1.5 h. Antibodies were visualized via DAB incubation for 10 min [24]. The images were collected and observed under an optical microscope (Mshot MF53, Guangzhou Mingmei Optoelectronics Technology Co., Ltd.).

### 2.5. Enzyme-Linked Immune Sorbent Assay (ELISA)

ELISA assay was conducted to detect serum TNF-*α*, IL-2, and IFN-*γ* of mice as per instructions of use (RUIXIN Bio-Tek). Briefly, ELISA kits were equilibrated at room temperature, 50 *μ*l of standard solution and sample were supplied to the sample plates and followed by the addition of 100 *μ*l of detection antibody, the well plate was sealed with sealing film, and cultured at 37°C for 60 min. 50 *μ*l substrate was provided to each well for culture in the dark at room temperature for 15 min. After incubation, stop solution at 50 *μ*l was supplemented to the wells, and the OD values at 450 nm were measured for each well.

The article "Metformin Synergizes with PD-L1 Monoclonal Antibody Enhancing Tumor Immune Response in Treating Non-Small Cell Lung Cancer and Its Molecular Mechanism Investigation" was retracted in 2023. Reasons: unreliable results or conclusions; concerns about the data; concerns about the peer review; concerns about the citations.

### 2.6. CD8+T Cells Isolation

The laboratory animals were sacrificed through cervical dislocation, and the spleens of mice were aseptically separated and placed in pre-cooled PBS solution, cut into pieces and repeatedly milled through a 200-mesh sterile copper mesh [25]. Cells were washed twice, centrifuged at 1200 rpm for 10 min, resuspended using RPMI 1640 medium with 100 *μ*L of calf serum, and counted. Mix the above cell suspension evenly, blend cell suspension with 0.2% trypan blue staining solution, count on a hemocytometer, and set the density at 8 × 10^6^ cells/mL. Cells were stained with PE-cy5 fluorescently labeled CD8 antibody using flow cytometry.

### 2.7. 3-(4,5-dimethylthiazol-2-yl)-2,5-diphenyltetrazolium bromide (MTT) Assay

Cells were cultured in 96-well plates containing 200 *μ*L/well, with three duplicate wells for each group of cells. The 96-well plate was transferred to an incubator (37 °C, 5% CO_2_), and then the cells adhere to the walls, the plate was treated with corresponding drugs as described above in grouping. After 24 hours, the plates were taken out, followed by the addition of 20 *μ*L 5 mg/mL MTT solution in each well and incubated in an incubator for 4 hours. The culture medium was carefully aspirated to terminate the culture. Following the supplement of 150 *μ*L dimethyl sulfoxide, the cells were placed on a shaker for 10 min to fully dissolve the purple crystals at a low speed [26]. The absorbance was detected at 490 nm via enzyme-linked immunosorbent assays (ELx800, Bio-Tek).

### 2.8. Co-Culture of CD8+ T Cells and LLC Cells

CD8+ T cells isolated by flow sorting were given with SIINFEKL peptide (10 ng/mL) and IL-12 (50 U/mL), treated for 24 h, washed, resuspended and cultured using RPMI 1640 medium containing IL-12 for 7 days to generate activated toxic lymphocytes. LLC cells were obtained from the Type Culture Collection, Chinese Academy of Sciences. The cells were incubated in DMEM containing 1% penicillin-streptomycin and 10% FBS at 37°C in a 5% CO_2_ incubator. LLC cells at 1.5 × 10^4^ cells/mL concentration were seeded in a 24-well plate and cultured in an incubator for 6 h. When the cells were completely adhered, the Transwell was placed in a 24-well plate, and CD8+T cells were transferred to a Transwell membrane (seeded CD8+T cell number was according to CD8+T : LLC = 10 : 1, 5 : 1, 4 : 1, 3 : 1, 2 : 1, 1 : 2) to establish Transwell co-culture system. According to the results of MTT detection, the optimal culture ratio was selected.

The article "Metformin Synergizes with PD-L1 Monoclonal Antibody Enhancing Tumor Immune Response in Treating Non-Small Cell Lung Cancer and Its Molecular Mechanism Investigation" was retracted in 2023. Reasons: unreliable results or conclusions; concerns about the data; concerns about the peer review; concerns about the citations.

### 2.9. Cell Grouping and Drug Delivery

CD8+ T cells and LLC cells were non-contact co-cultured at 2 : 1 ratio. The co-cultured cells were grouped into Control, metformin (3 mmol/L), PD-L1 MAb (1.5 *μ*g/ml), metformin combined with PD-L1 MAb group (metformin + PD-L1 MAb), Compound C (1 *μ*mol/L), metformin + Compound C, PD-L1 MAb combined with Compound C, and metformin combined with PD-L1 MAb and Compound C [27]. Cells were collected after 24 h for subsequent detection.

### 2.10. Statistical Analysis

GraphPad Prism version 9.0 (San Diego CA) was applied for statistical analysis. Data were merged from at least three biological and independent replicates and presented as mean ± standard deviation. The multivariant comparison was conducted using a one-way analysis of variance followed by Tukey's post hoc tests. The values of *P* < 0.05 were considered significant statistical differences.

## 3. Results

### 3.1. Metformin Combined with PD-L1 MAb Inhibits the Growth of Transplanted Tumors

After tumor cells were transplanted, tumor growth was observed every other day. The tumor was observed and measured using a vernier caliper every 3 days when the tumor grew to a measurable size. The mouse tumor of each group in vitro is exhibited in Figure 1(a). As shown in Figure 1(b), the body weight of mice generally is on the rise with the passage of time, and the body weight of the control increased the most. There was no evident difference in the growing trend of body weight among all drug treatment groups, however, the body weight growth of PD-L1 MAb and metformin + PD-L1 MAb increased greatest at 27 days than the rest. The tumor volume of mice in each group increased gradually over time. The fastest growth of tumors was revealed in the control, followed by the PD-L1 MAb treatment and metformin-treated group, and the increasing growth trend in metformin + PD-L1 MAb-treated group was the smallest (Figure 1(c)).

### 3.2. Metformin Combined with PD-L1 MAb Promotes CD8+TILs Infiltration

The volume growth trend of the transplanted tumor was measured, implying that metformin + PD-L1 MAb could effectively inhibit the growth trend of the transplanted tumor volume in mice. The expression of tumor proliferation signal Ki67 in tumor tissue was further detected by WB. The immunoblot band diagram is shown in Figure 2(a). Semi-quantitative was performed with *β*-actin as a reference. The expression of Ki67 was markedly decreased after drug administration as compared with the Control, and it was the lowest in metformin + PD-L1 MAb. However, no significant difference was revealed both in metformin and PD-L1 MAb treatment groups. The metformin + PD-L1 MAb treatment group was more effective in hindering the growth of xenograft tissue in mice than the metformin or PD-L1 MAb treatment alone that own the comparable ability to inhibit the growth of xenografts. Meanwhile, CD8 expression in tumor tissues was detected using immunohistochemistry and its phenotype was accessible as positive cells (Figure 2(b)). Compared with the control, the number of CD8+T cells increased after drug treatment and indicated strongly positive in the metformin + PD-L1 MAb group. The serum TNF-*α*, IL-2, and IFN-*γ* of mice were determined (Figure 2(c)). These functional cytokines were significantly increased in drug treatment, moreover, the previously described factors were the highest in metformin + PD-L1 MAb, followed by metformin.

The article "Metformin Synergizes with PD-L1 Monoclonal Antibody Enhancing Tumor Immune Response in Treating Non-Small Cell Lung Cancer and Its Molecular Mechanism Investigation" was retracted in 2023. Reasons: unreliable results or conclusions; concerns about the data; concerns about the peer review; concerns about the citations.

### 3.3. Metformin Combined with PD-L1 MAb Inhibits LLC Cells Viability in an AMPK Signaling Pathway-Dependent Manner

CD8+ T cells and LLC cells were co-cultured in a non-contact manner according to different cell ratios. The viability of co-cultured cells was detected in several ratios using MTT assays. The highest viability was observed when CD8+ T and LLC cells were co-cultured at 2 : 1 ratio (Figure 3(a)). As a potent, reversible, and selective AMPK inhibitor [28, 29], Compound C (BML-275) was added to inhibit AMPK activity in cell viability assays. As shown in Figure 3(b), each drug group can significantly inhibit the viability of LLC cells, especially metformin + PD-L1 MAb has the strongest power to inhibit LLC growth. After adding Compound C (1 *μ*mol/L), the efficiency of metformin and PD-L1 MAb in inhibiting LLC cell viability decreased, and the inhibitory power of metformin + PD-L1 MAb was also decreased. Metformin + PD-L1 MAb inhibited LLC cell growth dependent on the AMPK signaling pathway and could be inhibited by Compound C.

### 3.4. Metformin Combined with PD-L1 MAb Inhibits LLC Cells Proliferation via AMPK/mTOR

In addition to LLC cell viability experiments, in order to further study the dependence of metformin + PD-L1 MAb efficacy on the AMPK pathway, we used WB to detect p-AMPK and mTOR expression of CD8+ T cells in the co-culture system of CD8+ T cells and LLC cells. As presented in Figures 4(a)–4(c), metformin and metformin + PD-L1 MAb could increase the expression of p-AMPK while reducing that of mTOR in CD8+ T cells as compared to the control. Efficacy is AMPK-dependent and can be inhibited by Compound C. By activating the AMPK/mTOR pathway, cell substance synthesis and cell growth were inhibited to achieve anti-cancer effects. In addition, the expression of cell proliferation signal Ki67 in LLC cells was detected (Figure 4(d)). The expression of Ki67 in each drug group was greatly decreased, and that of Ki67 in metformin, PD-L1 MAb, metformin + PD-L1 MAb gradually decreased as compared with the control. After Compound C was added to the drug-treated group, the expression of Ki67 increased in each group.

The article "Metformin Synergizes with PD-L1 Monoclonal Antibody Enhancing Tumor Immune Response in Treating Non-Small Cell Lung Cancer and Its Molecular Mechanism Investigation" was retracted in 2023. Reasons: unreliable results or conclusions; concerns about the data; concerns about the peer review; concerns about the citations.

### 3.5. Metformin Combined with PD-L1 MAb Promotes CD8+T Cells to Secrete TNF-*α*, IL-2, and IFN-*γ*

Cell supernatants were collected after 24 h of treatment and ELISA was conducted to determine IL-2, TNF-*α,* and IFN-*γ* expression secreted by CD8+ T cells. The expression of the described factors was substantially increased in the drug-treated group, and maximum secretion was found in the metformin + PD-L1 MAb group (Figure 5). After Compound C inhibited the AMPK pathway, the capacity of CD8+ T cells to secrete TNF-*α*, IL-2, and IFN-*γ* was reduced, thereby making it an unavailable infiltrative environment for lung cancer cells.

## 4. Discussion

In the development of tumors, chronic stimulation of tumor antigens can promote the transformation of local CD8+TILs into central memory T cells (TCM) rather than effector memory T cells (TEM). TCM is affected by PD-1 and T cell immunoglobulin mucin-3 (Tim-3) and other depletion markers in the tumor immune microenvironment, and then resulting in immune depletion and loss of anti-tumor effect [30]. Metformin can downregulate the ratio of TCM/TEM by inhibiting the apoptosis of TEM cells, and inducing the transformation of immune-depleted TCM to activated TEM with anti-tumor effects that increase TNF-*α*, IL-2, and IFN-*γ* secretion and thereby inhibit immune depletion of CD8+TILs caused by continuous tumor antigen stimulation, enhance local infiltrating CD8+TILs both in number and activity [27].

Metabolites in the tumor microenvironment are of vital importance in tumor immune exhaustion [31]. Due to the altered blood supply and the energy imbalance of the tumor cells themselves, the tumor microenvironment has low concentrations of glucose and other metabolites, the interstitial pH is acidic, and the oxygen content is low [32]. Oxidative phosphorylation is necessary for the normal function of T cells. Therefore, tumor-infiltrating T cells lack the metabolites and energy required to perform effector functions. Recent researchers have found that metformin inhibits oxidative metabolism of tumor cells, changes the oxygen content of the tumor microenvironment, and then increases the oxygen supply of TILs, rescues T cells from the hypoxic environment, and enhances the killing effect of T cells [32, 33]. Since hypoxia is an important obstacle for tumor-infiltrating T cells to exert relevant functions, metformin can reconstruct a microenvironment available for tumor growth via oxidative metabolism regulation for tumor cells and release anti-tumor immune responses [34]. Therefore, when metformin is combined with immunotherapy, metformin can significantly improve anti-tumor immune function.

The article "Metformin Synergizes with PD-L1 Monoclonal Antibody Enhancing Tumor Immune Response in Treating Non-Small Cell Lung Cancer and Its Molecular Mechanism Investigation" was retracted in 2023. Reasons: unreliable results or conclusions; concerns about the data; concerns about the peer review; concerns about the citations.

PD-L1 can be used as an important immune checkpoint molecule, responsible for maintaining the body's immune balance and preventing the body's autoimmunity and tissue damage [35]. However, PD-L1 on the surface of tumor cells can bind to the PD-1 on the surface of activated cytotoxic T lymphocytes in tumor tissue, the inhibitory signal induced by PD-L1 can be inhibited, and the anti-cancer immunity of lymphocytes was inhibited. The tumor immune microenvironment is considered to be reversed if the PD-1/PD-L1 signaling pathway is blocked. Consequently, the effects of endogenous anti-tumor immune can be enhanced simultaneously. Furthermore, due to the highly expressed PD-L1 in tumor tissues, PD-1/PD- L1 may become an important target for immune therapy of tumors [36, 37].

We explore the efficacy of metformin and PD-L1 MAb in treating NSCLC at the animal and cell levels and study the effect of metformin combined with PD-L1 MAb against NSCLC. The results show that metformin + PD-L1 MAb is more effective in inhibiting the growth of transplantable cancer models and LLC cell viability than metformin or PD-L1 MAb alone. As previously demonstrated that metformin can inhibit the expression of PD-L1 in colon cancer HCT116 and SW480 cells [38]. Further, it is reported that metformin could reduce tumor cell PD-L1 expression and enhance anti-tumor immune response [39]. It can also downregulate PD-L1 by inhibiting IL-6 in esophageal squamous cell carcinoma, thereby promoting the anti-tumor immune response [40]. The above-reported studies may explain the reason why metformin combined with PD-L1 MAb has better anti-tumor efficacy than metformin or PD-L1 MAb-treated alone. The study also found that compared with the control, metformin, PD-L1 MAb, metformin + PD-L1 MAb inhibited tumor growth in cells and delayed proliferation of LLC cells in the co-cultured both CD8+ T and LLC cells. The expression level of the proliferation signal Ki67 in tumor tissues and cells was significantly reduced after drug treatment, and we also found that metformin + PD-L1 MAb inhibits tumor growth and proliferation better than metformin or PD-L1 MAb treatment alone. Immunohistochemical results showed that metformin + PD-L1 MAb increases CD8+ TILs in tumor tissue, reduces CD8+ T lymphocyte depletion, and enhances tumor immune response. ELISA was used to detect the cellular function factors TNF-*α*, IL-2, and IFN-*γ* in mice serum and cells. The secretion of TNF-*α*, IL-2, and IFN-*γ* was markedly increased in the drug group, and the secretion level of metformin + PD-L1 MAb was higher than that of metformin and PD-L1 MAb. IL-2 promotes differentiation and proliferation of T cells and B cells, effectively increases proliferation of TILs, inhibits tumor cell growth, and it also has a certain effect on malignant pleural effusion [41–43].

The article "Metformin Synergizes with PD-L1 Monoclonal Antibody Enhancing Tumor Immune Response in Treating Non-Small Cell Lung Cancer and Its Molecular Mechanism Investigation" was retracted in 2023. Reasons: unreliable results or conclusions; concerns about the data; concerns about the peer review; concerns about the citations.

Recent research has indicated a substantial increase in the number and activity of CD8+ TILs in tumor tissues after metformin treatment [44, 45]. Metformin has also been reported to inhibit primitive CD4+ T cell differentiation into Th1 cells and Th17 cells, thereby reducing IL-22 levels secreted by Th1 cells and Th17 cells, and blocking IL-22-mediated tumor proliferation and anti-apoptotic effects, has an important impact on the occurrence and development of tumors [46]. These effects depend on the AMPK-mTOR pathway. Metformin can activate AMPK, phosphorylate AMPK, and directly or indirectly inhibit its downstream mTOR, thereby inhibiting cell substance synthesis and cell growth, and achieving anti-cancer effects [47]. To further clarify relevant molecular mechanisms of metformin with PD-L1 MAb in treating NSCLC, we detected levels of p-AMPK and mTOR in CD8+ T cells and set up an AMPK inhibitor addition group (Compound C) to study whether metformin combined with PD-L1 MAb against NSCLC is dependent on the AMPK pathway. The results demonstrated that metformin combined with PD-L1 MAb could significantly inhibit the viability of LLC cells, increase the release of cytokines, and the expression of p-AMPK and mTOR in cells, and the results proved that the anti-tumor action of metformin with PD-L1 MAb on NSCLC was AMPK-dependent. However, the present study only verified the relationship between the anti-tumor mechanism of metformin combined with PD-L1 MAb and the AMPK pathway in LLC cell lines and has not been tested in other lung cancer cell lines. Second, it is limited to the preliminary discussion of the molecular mechanism, the anti-tumor mechanism investigation of metformin combined with PD-L1 MAb is deeply needed.

## 5. Conclusions

Taken together, this study demonstrated that metformin synergized with PD-L1 MAb increased the infiltration capacity of CD8+ T cells, enhanced tumor immune response, and had better efficacy in the treatment of NSCLC than metformin or PD-L1 MAb. And its anti-tumor mechanism might link to the inhibition of either AMPK pathway activation or directly inhibiting mTOR. The results of the current research provide an experimental foundation for the application of anti-PD-L1 antibody combined with metformin against NSCLC, as an alternative management option for NSCLC.

The article "Metformin Synergizes with PD-L1 Monoclonal Antibody Enhancing Tumor Immune Response in Treating Non-Small Cell Lung Cancer and Its Molecular Mechanism Investigation" was retracted in 2023. Reasons: unreliable results or conclusions; concerns about the data; concerns about the peer review; concerns about the citations.

## Figures and Tables

**Figure 1:** The tumor growth of mice of lung cancer subcutaneously transplanted tumor. (a) The xenograft tumor growth of each group: metformin, PD-L1 MAb, metformin + PD-L1 MAb and Control. The mice body weight (b) and xenograft tumor volume (c) was quantified (*n* = 6).

**Figure 2:** The xenograft tumor tissue cells' proliferation, immune and inflammation in LLC cells xenograft tumor mice. (a) Ki67 expression in xenograft tumor tissue detected by WB. (b) CD8+ antibody in tumor tissue of LLC cells xenograft tumor mice. CD8+ positive cells were colored in brown (magnification = 400x). (c) Serum IL-2, TNF-*α,* and IFN-*γ* in LLC cells of xenograft tumor mice. Multiple group comparisons applied ANOVA and Tukey's post hoc tests. ^#^, *P* < 0.05; ^##^, *P* < 0.01 vs Control.

**Figure 3:** Viability of co-cultured CD8+ T and LLC cells. (a) Cell viability of different ratio of co-cultured CD8+ T and LLC cells. (b) Cells viability was detected by MTT assay. CC, Compound C (AMPK inhibitor). Multiple group comparisons applied ANOVA and Tukey's post hoc tests. ^#^, *P* < 0.05; ^##^, *P* < 0.01 vs Control.

**Figure 4:** Inhibited LLC cells proliferation in metformin combined with PD-L1 MAb. (a) p-AMPK, mTOR, and Ki67 protein expression were detected by Western blot. Relative p-AMPK (b) and mTOR (c) expression in CD8+T cells were calculated based on the *β*-actin. (d) Ki67 expression in LLC cells was quantified. Multiple group comparisons applied ANOVA and Tukey's post hoc tests. ^#^, *P* < 0.05; ^##^, *P* < 0.01 vs Control.

**Figure 5:** Serum IL-2, TNF-*α,* and IFN-*γ* level in CD8+T cells were detected using ELISA assays. Multiple group comparisons applied ANOVA and Tukey's post hoc tests. ^#^, *P* < 0.05; ^##^, *P* < 0.01 vs Control.

## Data Availability

The data supporting the findings of this study are available from the corresponding author.
